The article "Tensiomyography and Statistical Analysis Based Muscle Change Detection in Multiple Sclerosis for Smart Healthcare" was retracted in 2023. Reasons: signs of a paper mill; suspected computer-generated content; unreliable results or conclusions; lack of ethics approval or compliance.

# Tensiomyography and Statistical Analysis Based Muscle Change Detection in Multiple Sclerosis for Smart Healthcare

**DOI:** 10.1155/2022/5225851

**Published:** 2022-12-02

**Authors:** Ligia Rusu, Marius Cristian Neamtu, Oana Maria Neamtu, Mihai Robert Rusu, Mihnea Ion Marin, Daniel Danciulescu, Jude Hemanth

**Affiliations:** ^1^Sport Medicine and Physical Therapy Department, University of Craiova, Craiova 200585, Romania; ^2^Physiology Department, University of Medicine and Pharmacy Craiova, Craiova 200349, Romania; ^3^Applied Mechanic Department, University of Craiova, Craiova 200585, Romania; ^4^Department of ECE, Karunya Institute of Technology and Sciences, Coimbatore, India

## Abstract

The impact of demyelinization on muscle fiber changes and the type of changes in multiple sclerosis (MS) is very hard to estimate. One of the major problems of MS patients is muscle fatigue and decrease of muscle force in the range of 16–57%. The objective of this research work is to estimate various aspects of muscle changes at tibial muscle (mTA) level using a noninvasive method named as tensiomyography (TMG). TMG provides information about muscle functions in MS. This study includes 40 MS patients among which 18 are males (45%) and 22 are females (55%). They are divided in two subgroups: subgroup A and subgroup B. Subgroup A includes 20 MS patients without clinical decelable gait disorders and subgroup B includes 20 MS patients with clinical decelable gait disorders. Also, we have a control group that includes 20 healthy people with the same average age. Average age is 38.15 ± 11.19 y for MS patients and 39.34 ± 10.57 for healthy people. Evaluation measures include ADL score and EDSS scale. The ADL score is 0 for patients from subgroup A and 1 for patients from subgroup B. The EDSS score is 1 for subgroup A and 2.5 for subgroup B. This study confirms the importance of TMG based evaluation of muscle changes in MS patients. This smart healthcare system is also used for prediction of the muscle changes and muscle imbalance. Contraction time (Tc) recordings are used to detect the muscle fatigue which is a specific symptom of MS. The value of Tc for subgroup A is 45.8 ms and subgroup B is 61.37 ms for right side. Analysis of these two parameters such as Dm and Tc could define the muscle behaviour and help provide early information about the possibility of developing gait disorders. This smart TMG system analyses the muscle tone in the best possible way to predict the onset of any diseases which is an integral part of the smart healthcare system.

## 1. Introduction

Multiple sclerosis (MS) is an autoimmune disease which affects myelin that surrounds nerve cell axons. The result of the demyelinization process is specific for MS which leads to the development of the local inflammation and subsequently the installation of scars nerve cell axons. This results in the decrease of nervous conductibility. This is the main reason for the sensor-motor difficulties in MS patients. However, the demyelinization process is very complex and nonlinear. It is very difficult to estimate the intensity of muscle fiber changes and the type of changes. Several researchers have analyzed the decrease of muscle force with the isokinetic system which leads to muscle atrophy [1, 2]. Specifically, lower limb muscles are much affected than the upper limb muscles [3].

One of the major problems for MS patients is muscle fatigue and decrease of muscle force that could be between 16 and 57% [4]. The main reason seems to be the demyelinization process at the upper central neuron [5]. Accordingly, muscle activation in MS is reduced because of the deficiency in motor units [4]. Other observations are the decrease in the production of peripheric nervous mediators, reduction in the dimensions of muscle fibers, change of muscle types fibers distribution, and neuromuscular transmission. Muscle changes-based research in MS also includes muscle biopsy at vastus lateral muscle. MS patients with EDSS score of 4.75 show the presence of type II-a myosin heavy chain (MHC) isoform. This increases in according with the disability level and is associated with decrease of muscle fiber type I.

Thus, fibers from the MS group displayed a subtle shift in fast MHC isoform coexpression and a modest reduction in cross-bridge number, density, or average force. All these occurs with no change in maximal cross-bridge cycling rate or susceptibility to intracellular metabolites. These changes explain the part of the muscle weakness and fatigue experienced by individuals with MS [6]. MS patients seem to have a lower percentage of type I fiber and a higher percentage of type II fiber. Changes in muscle fibers distribution are connected with spasticity and muscle weakness which are seen in most of the MS patients. In spite of the availability of many literature on spasticity, the necessity for more information still persists for the assessment of muscle weakness in MS. Muscle weakness is one of the main features that disturbs the muscle force which impacts the daily activities of human beings.

## 2. Related Works

In this context, there are a lot of studies that discuss about correlation between muscle weakness in MS and the MMT scale (manual muscle testing) based estimated muscle force values. McDonald and Compston, in their book McAlpine's Multiple Sclerosis [7], show that from a group of 301 patients, 52% suffer from muscle weakness. Hoang et al. demonstrates the presence of muscle weakness among 72% patients from a total of 142 patients with MS [8].

At the same time, muscle weakness in MS is associated with decrease of fitness, functional status [9, 10], and general fatigue [9]. This leads to decrease in the level of daily activities and also the quality of life. Thus, it is evident that the muscle fiber dimension reduction is the major element in the development of muscle weakness.

Literature survey describes numerous pathogenic mechanisms which are the reasons for the evolution of unpredictable nature of lesion evolution in MS patients. The unpredictability is mainly due to the presence of older lesions and new lesions at the same time. This indicates the dynamic evolution of these diseases and the nonlinear changes in the progression of this disease. Silent lesions are a specific feature and pathognomonic for MS [11]. In the context of evolution of MS, clinical evaluation is the first process and it is followed by analysis of cerebrospinal fluid. Thus, it is necessary and possible to have the evolution pattern of immune response. Evoked potential and MRI also assist in the complete diagnosis [12].

Evoked potential includes visual auditive and somatosensorial potentials for assessing the magnitude and response time after stimulation. These potentials provide a clear picture about nervous central system status functionality. The advancement in smart healthcare systems aid in the identification, development, and implementation of a new model for data acquisition for early diagnosis, monitoring, and treatment planning. The aim of this paper is to present various aspects of muscle changes at tibial muscle (mTA) level using a noninvasive method named tensiomyography (TMG) which gives us numerous information about muscle function in MS. The rationale of this study is to present some aspects regarding the possible muscle changes produced in MS with a technology like TMG. This will assist in detecting the onset of any gait disorders developed during the MS. Analysis of the muscle response after electrical stimulation with TMG provides information about the muscle fibers' response in terms of muscle fatigue. Early detection of gait abnormalities is extremely important for proper treatment planning.

The rest of the paper is organized as follows: Section 3 deals with the materials and methods, Section 4 demonstrates the statistical analysis carried out on the real-time data, Section 5 illustrates the experimental results and discussion, and Section 6 provides the conclusions with the key findings of this real-time research work.

## 3. Materials and Methods

The study includes 40 MS patients among which are 18 males (45%) and 22 females (55%). The control group includes 20 healthy people with the same average age for the comparative analysis of TMG parameters. However, the analysis is always complex due to the polymorphism of lesions in MS and the clinical and functional evolution. The criteria for selection of MS patients are certainty of MS diagnosis in accordance with clinical and paraclinic criteria and clear evidence for not associated with any other pathologies. Diagnosis criteria [13–15] that are accounted for in this work are as follows: certainty of MS, minimal two episodes of clinical manifestation of MS, clinical symptoms for two separately different lesions or clinical symptoms for one clinical lesion, and another subclinical lesion that is demonstrated by neurophysiologic evaluation or MRI. The exclusion criteria of this research work are lack of all clinical information about the patient and the patients that do not agree to participate in the study.

The small number of the patients is mainly because of the huge diversity in the evolution of the MS in different moments, difficulty in generating the evolution of symptomatology, and difficulty in ambulation. The patient's selection is based on gender, age, and evolution stage because of the requirement for the variety of abnormalities. However, MS is more frequent in female patients. Additionally, the following aspects are considered:

- All patients are from urban zone
- Average age is 38.15 ± 11.19 y for MS patients and 39.34 ± 10.57 for healthy people
- Subgroup A consists of 20 MS patients without clinical decelable gait disorders
- Subgroup B consists of 20 MS patients with clinical decelable gait disorders

Analysis of gait disorders from the clinical point of view is made using ADL scale [16]. The interpretation is given as follows: 0 = normal (8 points); 1 = mild disability (6 points); 2 = moderate disability (4 points); 3 = severe disability (less than 4 points). Patients from subgroup A have ADL score 0, and patients from subgroup B have ADL score 1. For functional evaluation, we use EDSS scale which has a score from 0 to 10. The score is 1 for subgroup A and 2.5 for subgroup B. For subgroup A, Tc value is 60.3 ms for left side and 45.8 ms for right side. For subgroup B, Tc value is 61 ms for left side and 61.375 ms for right side. For subgroup A, Dm value is 3.2 mm for left side and 3.9 mm for right side. For subgroup B, Dm value is 3.83 mm for left side and 3.69 mm for right side. We observe a significant difference for both subgroups in terms of Tc and Dm.

Tensiomyography is a new method for the assessment of the muscle functional status which allows to evaluate the contractile proprieties of muscle fibers after electrical stimulation. The assessment includes tibial anterior muscle (mTA) and analysis of two TMG parameters: muscle displacement (Dm) and time of contraction (Tc) during electrical stimulation. These parameters are correlated with muscle fatigue and muscle composition of type I and type II muscle fibers. The statistical analysis is focused on data distribution, descriptive analysis, and analysis of significant variance (*p* < 0.05) between MS subgroups and control group. Results show normal distribution of the data and significant differences between TMG parameters that includes decrease of Dm and increase of Tc for subgroups A and B in comparison to the control group.

The method consists of application of a progressive electrical stimulation (single stimulation but progressive increase of intensity), using surface electrodes, from 10 mA until the muscle response becomes maximal. An illustration on muscle contraction is given in Figure 1. The stimulation consists of successive impulses and the frequency of stimulation is 5–25 Hz, 40–50 V. Time of stimulation is 10 s. The muscle response is collected by a sensor of TMG (G40, RLS Inc.), which is placed on the maximal muscle belly point. The exact point is detected by maximal isometric contraction in rest position before stimulation. The surface electrodes are placed towards the sensor. The stimulus is applied on the proximal electrode. The electrical stimulation generates isometric muscle contraction. The sensor has a bow of size 0.17 N/mm and is placed perpendicular to the muscle surface.

The electrical stimulation produces a transversal displacement of muscle fibers which is taken over by the sensor. The displacement is proportional to the muscle force during isometric contraction. By this way, displacement and other TMG parameters can help assess the muscle fatigue. Measure of muscle response, database, and analysis of the recording data are made using a dedicated TMG software.

The TMG parameters are as follows:

- Delay time (Td): the time elapsed from the moment of stimulation to the level of reaching 10% muscle contraction (ms);
- Contraction time (Tc): the time between the moment when the muscle contraction is 10% and muscle contraction is 90% from maximal level (ms).
- Contraction time depends on muscle composition (percent of type I fiber and type II fiber). The Tc increases if the percent of type II fibers increase and type I fibers decrease and this is in correlation with the onset of muscle fatigue.
- Sustain time (Ts): the time between the moment when the contraction is 50% and the moment when the relaxation reaches 50% (ms);
- Relax time (Tr): the time elapsed from the moment when the relaxation is 50% and the moment when the relaxation is 90% (ms);
- Amplitude of muscle displacement Dm (mm) is correlated with Tc and depends on muscle tissue elasticity. Dm increases during muscle explosive force and decreases if the muscle tone increases.

In this work, the analysis is performed only with two parameters Dm and Tc. These two parameters allow estimating the muscle composition and behaviour of muscle fatigue. The muscle fatigue is correlated with Tc and Dm. The assessment of tibial muscle mTA (Figure 2) is given much emphasis because this muscle is involved in foot dorsal flexion during the first moment of the gait.

## 4. Statistical Analysis

The aim of the statistical analysis is to identify the significant differences of Dm and Tc between the control group and subgroups of MS patients. The statistical analysis is also used for evaluating the significant differences from left and right side, for each subgroup A and B. This is to assess the functional asymmetry and muscle imbalance. Data analysis-based software packages are used for the statistical analysis.

A database is initially created with the experimental data from the significant aspects for this research which are extracted. The recording values of the parameters are analyzed to visualize the variables, and the statistical analysis is performed to observe the significant differences between data series for each group. Descriptive data (means SD) are reported for the entire patient cohort. Normal distribution is tested using the JB (Jarque–Bera) test and visual analysis of Gauss function for Dm and Tc.

The Jarque–Bera test is the easiest way to test the assumption that the values in a dataset are normally distributed. This test uses the following hypotheses: *H*_0_: the data are normally distributed; *H*_1_: the data are not normally distributed.

We apply the *t*-test for equal and unequal variances depending on the results of the Levene test, for Dm and Tc.

Levene's test is an inferential statistic used to assess the equality of variances for a variable calculated for two groups. Levene's test is used before a comparison of means. The *t* test is a statistical test that is used to compare the means of two groups. It is used in hypothesis testing to determine two groups that are different from one another from the TMG parameters. Statistical significance is set at a level of *p* < 0.05.

## 5. Experimental Results and Discussion

The normalization of the measurements for all three groups (control, subgroup A, and subgroup B) is checked using the Jarque–Bera test (JB test).  Table 1 shows the analysis of Gauss function for Dm and Tc.

Statistical significance is set at a level of *p* < 0.05. It is evident from the table that all data follow normal distribution. Gauss graphics are presented in Figures 3–5 and the normal distribution is followed in them too.

Table 2 shows the average values and SD of Tc and Dm for mTA. This falls under the category of descriptive statistical analysis.

We observe in Table 2 that Dm are mostly with small values which are close for both subgroups A and B (subgroup A 3.9 mm and subgroup B 3.69 mm) for the right side. The values are lesser than those for the control group where a value of 5 mm is observed for Dm of the right side. The differences between MS subgroups and control group are also significant for the left side. The Dm values are almost similar for subgroups A and B (subgroup A 3.2 mm and subgroup B 3.83 mm). The Dm value of the control group is 4.5 mm. Tc parameters are observed with higher values for subgroups A and B, but with a significant difference between the subgroups as shown in Table 2. The value of Tc for subgroup A is 45.8 ms and subgroup B is 61.37 ms for right side. The values are lesser than the values for the control group whose value is 42.78 ms.

However, higher values are observed for the left side for both subgroups A and B. The values are also similar with subgroup A recording a value of 60.3 ms and subgroup B recording a value of 61 ms. The values are higher than the values for the control group whose value is 41.85 ms. An analysis on the variation of Dm and Tc for subgroups A and B is carried out to check if there are any significant differences between subgroups and control group. The *t*-test based on series dispersion, equal, or unequal variances is used as the statistical method for this analysis. Tables 3 and 4 show the results of the Levene test which provides information about the type of dispersion.

Based on the above results, the *p* value is estimated to quantify the significance of the variance. These details are supplied in Tables 5–7.

A significant difference between two subgroups A and B for both parameters is observed, which is constant for both parameters. Also, significant differences between subgroups and control group for both parameters are also observed from Tables 5 and 6. An analysis is also performed for the estimation of functional symmetry (right/left) for each subgroup and the results are presented in Table 7. A significant difference is observed for Tc parameters and only for subgroup A (*p*=0.025).

Analysis of the results in this research reveals that the average Dm values are smaller for subgroups A and B in comparison to the average values for the control group. This means that the patients from subgroups A and B have an increase of muscle tone. Tc is higher for MS patients, and it is correlated with muscle fibers type. This provides information about the decrease in the percent of muscle type I fibers and increase in the risk of muscle fatigue. Increase in the percent of muscle type II fibers is correlated with small values of Dm which indirectly indicates the increase in muscle tone. Motor performances of lower limb depend on the muscle proprieties. TMG assists in assessing the muscle changes from the morphofunctional point of view in MS patients. Muscle tone and muscle force are components that depend on the muscle composition and muscle atrophy. Muscle atrophy is often visible in MS patients, which is evidence for the onset of muscle imbalance.

The small values of Dm in MS and the values of Dm for subgroup A explain the nondecelable clinical gait disorders of subgroup A. This aspect is related with the ankle kinetic during the gait and it is an important element for initiation of the gait. In subgroup B, the average value for Dm is very less than the values of the control group. This is the main reason for the gait disorders to be clinically complex between subgroups A and B. Tc parameter values are higher and this suggests an increase of muscle fibers type II. This could be considered like an adaptive process during the pathology of MS. This aspect was also observed by Kent-Braun et al. [17] in their study. At the same time, muscle biopsy of mTA revealed the decrease in the percent of type I fibers and increase in type II fibers in MS patients. This new muscle configuration is called as “fiber effect” and is based on fibril IIx (transition fibers). It also depends on the morphofunctional muscle changes and requirements.

Most of the research works have focused only on muscle changes during spasticity in stroke. In our research, more emphasis is given for the assessment using TMG for MS patients. This is the main contribution of the work. The proposed model is in contrast to the study of Krizaj et al. [18] which analyses the TMG parameters (Tr, Ts, Dm) in stroke for monitoring the effect of botulin toxin BTX-A administration. This study confirms the importance of TMG in the assessment process of muscle changes in MS, monitoring the evolution and the prediction of the muscle changes and muscle imbalance. Based on the study of Šimunic et al. [19], this work can be extended in future to propose the rehabilitation process in athletes in terms of muscle fatigue.

## 6. Conclusions

A smart healthcare system is heavily dependent on the smart diagnostics methodologies. In this research work, the smart sensor based TMG system is used to detect the muscle strength, which can be used to predict the gait disorders and other MS abnormalities. The smart assessment is based on Tc and Dm. Contraction time Tc is high for mTA, and it is correlated with increase of type II fibers and muscle fatigue which are specific symptoms of MS. TMG is a noninvasive way for assessment of the muscle proprieties without involving the tendon property or joint movement during the electrical stimulation. Analysis of these two parameters such as Dm and Tc can define the muscle behaviour and help to have early information about the possibility of developing the gait disorders. Hence, the therapeutic intervention can be started early to limit the progression of muscle damage and activate the neuroplasticity mechanism. Dm parameter is also useful for monitoring the spasticity and prediction of muscle tone evolution that can disturb the lower limb function. TMG is possible for monitoring the evolution of muscle (mTA) behaviour during and in time and could help for evaluating the effect of therapeutic intervention applied for maintaining the functional muscle status in MS.

## Figures and Tables

**Figure 1:** Graphic of muscle displacement (and other TMG parameters) during electrical stimulation.

**Figure 2:** Position of the electrodes and sensor on the mTA.

**Figure 3:** Control group Gauss function: (a) Dm; (b) Tc.

**Figure 4:** Subgroup A Gauss function: (a) Dm; (b) Tc.

**Figure 5:** Subgroup B Gauss function: (a) Dm; (b) Tc.

**Table 1:** Jarque–Bera test and *p* value^*∗*^ for Dm and Tc.

JB test	m TA right side		m TA left side	
	Tc (ms)	Dm (mm)	Tc (ms)	Dm (mm)
JB test control group	1.548	1.465	1.270	1.270
*P* value control group	0.461	0.481	0.530	0.530
JB test group A	3.012	2.970	1.117	0.988
*P* value group A	0.222	0.227	0.572	0.610
JB test group B	0.055	0.041	6.016	1.208
*P* value group B	0.973	0.979	0.054	0.547

^*∗*^Statistical significance was set at a level of *p* < 0.05.

**Table 2:** Average values and standard deviation (SD) for Dm and Tc, for m TA.

Group		Dm (mm)		Tc (ms)	
		Right	Left	Right	Left
Control group	Average	5	4.5	42.78	41.85
	SD	2.1	2.2	10.69	11.70

MS without gait disorders (subgroup A)	Average	3.9	3.2	45.8	60.3
	SD	2.3	2.3	22.57	22

MS with gait disorders (subgroup B)	Average	3.69	3.83	61.375	61
	SD	1.45	1.91	14.82	18

**Table 3:** Result of the Levene test for Tc.

TA muscle	Subgroups A-B	Control group − subgroup A	Control group − subgroup B
Right	*t*-UV	*t*-UV	*t*-EV
Left	*t*-UV	*t*-UV	*t*-EV

*t*-UV, *t*-test unequal variances; *t*-EV, *t*-test equal variances.

**Table 4:** Result of the Levene test for Dm.

TA muscle	Subgroups A-B	Control group − subgroup A	Control group − subgroup B
Right	*t*-EV	*t*-UV	*t*-EV
Left	*t*-EV	*t*-EV	*t*-EV

*t*-UV, *t*-test unequal variances; *t*-EV, *t*-test equal variances.

**Table 5:** *P* value^*∗*^ (test t-Student) for Tc, compare subgroups A and B, compare subgroups and control group.

TA muscle	Subgroups A-B	Control group − subgroup A	Control group − subgroup B
Right	0.008	0.034	0.00038
Left	0.044	0.01	0.0001

^*∗*^Statistical significance was set at a level of *p* < 0.05.

**Table 6:** *P* value^*∗*^ (test t-Student) for Dm, compare subgroups A and B, compare subgroups and control group.

TA muscle	Subgroups A-B	Control group − subgroup A	Control group − subgroup B
Right	0.046	0.044	0.013
Left	0.047	0.017	0.0182

^*∗*^Statistical significance was set at a level of *p* < 0.05.

**Table 7:** *P* values^*∗*^ (test t-Student) for Dm and Tc, functional symmetry right/left.

TA muscle	Right/left − subgroup A	Right/left − subgroup B
Tc	0.025	0.485
Dm	0.158	0.210

^*∗*^Statistical significance was set at a level of *p* < 0.05.

## Data Availability

There are no data associated with this research work.

## References

[1] Dalgas U., Stenager E., Ingemann-Hansen T. (2008). Review: multiple sclerosis and physical exercise: recommendations for the application of resistance-endurance- and combined training. *Multiple Sclerosis*.

[2] Sandoval A. E. (2013). Exercise in multiple sclerosis. *Physical Medicine and Rehabilitation Clinics of North America*.

[3] White L. J., McCoy S. C., Castellano V. (2004). Resistance training improves strength and functional capacity in persons with multiple sclerosis. *Multiple Sclerosis*.

[4] Ng A. V., Miller R. G., Gelinas D., Kent-Braun J. A. (2004). Functional relationships of central and peripheral muscle alterations in multiple sclerosis. *Muscle & Nerve*.

[5] Jorgensen L. M., Nielsen J. E., Ravnborg M. (2005). MEP recruitment curves in multiple sclerosis and hereditary spastic paraplegia. *Journal of the Neurological Sciences*.

[6] Garner D. J. P., Widrick J. J. (2003). Cross-bridge mechanisms of muscle weakness in multiple sclerosis. *Muscle & Nerve*.

[7] Miller D., McDonald I., Compston A., Compston A., Confavreux C., Lassmann H. (2006). Chapter 9 - multiple sclerosis in the individual and in groups: a conspectus. *McAlpine’s Multiple Sclerosis*.

[8] Hoang P. D., Gandevia S. C., Herbert R. D. (2014). Prevalence of joint contractures and muscle weakness in people with multiple sclerosis. *Disability & Rehabilitation*.

[9] Chung L. H., Remelius J. G., Van Emmerik R. E. A., Kent-Braun J. A. (2008). Leg power asymmetry and postural control in women with multiple sclerosis. *Medicine & Science in Sports & Exercise*.

[10] Thoumie P., Lamotte D., Cantalloube S., Faucher M., Amarenco G. (2005). Motor determinants of gait in 100 ambulatory patients with multiple sclerosis. *Multiple Sclerosis Journal*.

[11] Lassmann H. (2001). Classification of demyelinating diseases at the interface between etiology and pathogenesis. *Current Opinion in Neurology*.

[12] Noseworthy J. H., Lucchinetti C., Rodriguez M., Weinshenker B. G. (2000). Multiple sclerosis. *New England Journal of Medicine*.

[13] Hufschmidt A., Lücking C. H. (2002). *Neurologie integrală de la simptom la tratament*.

[14] Eleiwy J. A. (2021). Characterizing wavelet coefficients with decomposition for medical images. *Journal of Intelligent Systems and Internet of Things*.

[15] Abdulazeez A. M. (2021). Ultrasound medical images classification based on deep learning algorithms: a review. *Fusion: Practice and Applications*.

[16] Williams B. C., Fries B. E., Foley W. J., Schneider D., Gavazzi M. (1994). Activities of daily living and costs in nursing homes. *Health Care Financing Review*.

[17] Kent-Braun J. A., Ng A. V., Castro M. (1997). Strength, skeletal muscle composition, and enzyme activity in multiple sclerosis. *Journal of Applied Physiology*.

[18] Krizaj D., Grabljevec K., Šimunic B. Evaluation of muscle dynamic response measured before and after treatment of spastic muscle with a BTX-A: a case study.

[19] Šimunic B., Pišot R., Djordjevic S., Kugovnik O. Age related changes of the skeletal muscle contractile properties.

